# Study on the Efficacy of Electric Acupuncture in the Treatment of Premature Ejaculation Based on Testosterone Level

**DOI:** 10.1155/2022/8331688

**Published:** 2022-03-22

**Authors:** Xiangpeng Lu, Hao Han, Zhibiao Zhang, Hao Chen, Xingru Huang, Rui Zhang

**Affiliations:** ^1^The Second Affiliated Hospital of Heilongjiang University of Chinese Medicine, Heilongjiang, China; ^2^Heilongjiang Traditional Chinese Medicine Hospital, Heilongjiang, China

## Abstract

**Objective:**

To investigate the clinical efficacy and possible mechanism of electroacupuncture in the treatment of premature ejaculation.

**Methods:**

50 cases of premature ejaculation patients who met the diagnostic criteria were randomly divided into 2 groups with 25 cases in each group. The observation group was treated with electroacupuncture, and the control group was treated with Longdan Xiegan decoction. The treatment period was 4 weeks. Ejaculation latency (IELT), sexual satisfaction score of patients, sexual satisfaction score of partners, testosterone test, and drug safety assessment were performed in all 4 groups before and after treatment.

**Results:**

IELT was prolonged in all groups after treatment, the difference was statistically significant (*P* < 0.05). At the same time, the IELT of the observation group was significantly higher than that of the control group after treatment. Life satisfaction scores of patients and spouses in 2 groups were improved after treatment compared with before treatment, the difference was statistically significant (*P* < 0.05). After treatment, the satisfaction scores of patients and spouses in the observation group were higher than those in the control group, and the difference was statistically significant (*P* < 0.05). Before treatment, there was no significant difference in serum testosterone levels among all groups (*P* > 0.05). Serum testosterone levels in all groups were decreased after treatment compared with before treatment, with statistical significance (*P* < 0.05). After treatment, the serum testosterone level of the observation group was lower than that of the control group, and the difference was statistically significant (*P* < 0.05). During the treatment, the adverse reactions in each group disappeared after treatment, and no obvious abnormality was observed in the safety indicators.

**Conclusion:**

Electroacupuncture can improve the symptoms of premature ejaculation, which may be related to the regulation of serum testosterone by acupuncture.

## 1. Introduction

Premature ejaculation (PE) is a common disease in male sexual dysfunction, and its incidence rate is very high. PE refers to conditions in which the penis has not been inserted into the vagina, the parties have not contacted or have just been exposed to ejaculation, or ejaculation in less than 1 minute after insertion, resulting in an inability to perform normal sexual intercourse for more than 1 month. This disease is a common sexual dysfunction disease in adult men, and data show that about 75% of men will have premature ejaculation in their lifetime [1]. Among adult males, the incidence rate is 35%–50% [2]. Under the pressure of modern stressful life pace, the incidence rate of male premature ejaculation is on the rise every year, which greatly reduced the happiness in family.

At present, the treatment methods of Western medicine include psychotherapy and behavioral intervention, the application of antidepressants, the use of drug local anesthesia, and surgical treatment. Traditional Chinese medicine has a long history of treating the disease, accumulated rich clinical experience, and achieved good clinical efficacy. In traditional Chinese medicine, there are mainly traditional Chinese medicine, acupuncture, moxibustion, massage, umbilical therapy, acupoint application, acupoint embedding, and other relatively conservative treatment methods [3].

With the modern tense pace of life, physical overdraft, life pressure, air, food, and water pollution, and other factors, the incidence of male premature ejaculation has been increasing year by year, greatly affecting the quality of life of the couple and family happiness and stability. Now, there are many methods to treat premature ejaculation, and the application of antidepressants easily increases the misunderstanding of patients and increases the psychological burden. The curative effect of surgical therapy is not exact, and the harm is great. Psychological or behavioral treatment is difficult to operate clinically, long-term use of local anesthetics may cause erectile dysfunction, and to a certain extent, the internal environment of the woman has certain damage, affecting life. The operation of acupuncture and moxibustion is simple, and the deputy general use is small. Therefore, this study explores the efficacy of electroacupuncture in the treatment of premature ejaculation.

The etiology of premature ejaculation is complex, and the treatment is mainly based on serotonin reabsorption inhibitors. Studies have shown that low doses of testosterone combined with doxazosin in the treatment of premature ejaculation can achieve satisfactory results [4]. This study investigated 50 patients with premature ejaculation and observed the changes of IETE and spouse satisfaction and testosterone level in the two groups after treatment, which will provide more effective treatment methods for clinical application.

## 2. Methods

### 2.1. Ethical Statements

The included cases were from the outpatient department of acupuncture and moxibustion in our hospital from January 2019 to June 2021. The 50 patients who met the criteria for case selection were numbered from 1 to 50 according to the order of medical treatment. The odd and even numbers were divided into electroacupuncture group (hereinafter referred to as the observation group) and control group, with 25 patients in each group. All patients wrote the informed consent, and these studies were approved by the ethics boards of the hospital.

### 2.2. Diagnostic Criteria

“Chinese traditional medicine new medicine clinical research guiding principle” for premature ejaculation in Chinese medicine diagnosis standard was referred: during sexual intercourse, ejaculation when the penis has not been inserted into the vagina, or when both sides have not been contacted or just contacted, or ejaculation in less than 1 minute after inserting, as a result cannot have normal sexual intercourse, and lasting for more than 1 month are the diagnostic criteria for this disease. Inclusion criteria are as follows: (1) the patients meet the above diagnostic criteria for premature ejaculation; (2) age ≥24 years and ≤48 years and course of disease >3 months and <10 years; (3) married or with a regular sexual partner and sexual life for more than half a year; (4) no surgical treatment was performed; (5) patients who have not taken drugs or received other treatments recently (within 1 month before the treatment); and (6) voluntarily participate in the clinical study and signed informed consent.

Exclusion criteria are as follows: (1) ejaculation latency >1 min; (2) persons aged <24 or >48; course of disease ≤1 month or ≥10 years; (3) the penis and testicles have organic lesions, including phimosis, foreskin too long, foreskin frenulum too short, and cryptorchidism; (4) inflammation of the genitourinary system, such as prostatitis, seminal vesiculitis, vermontanetis, epididymitis, spermatic cord quietly varicose, and urethritis; (5) hyperthyroidism; (6) schizophrenics; (7) erectile dysfunction; (8) patients with abnormal blood lipid, blood glucose, and blood pressure; (9) patients with other diseases of brain, heart, liver, and kidney that affect the effectiveness evaluation of this treatment; (10) patients with neurological diseases (brain tumor, cerebrovascular disease, and spinal cord injury); (11) patients who have taken drugs or received other treatments recently (within 1 month before the treatment); (12) irregular sexual life; (13) the patient had undergone surgical treatment; and (14) needle sickness.

### 2.3. Treatment

The observation group was treated in the acupuncture points: Zhongji point (−) and Sanyinjiao point (+). The frequency was 2–100 Hz, the current intensity was 0.1 mA–1.0 mA, and the intensity was tolerated by patients with slight local beating. The needle was left for 30 min. Once a day, 6 times in a row, then rest for 1 day, 6 times in a course of treatment, a total of 4 courses. The control group was given one dose of Longdan Xiegan decoction every day, 300 ml of decoction, twice in the morning, and 1 hour after dinner.

### 2.4. Observation of Curative Effect Index

The changes of IELT before and after treatment were observed, and the average value of three sexual lives before and after treatment was taken as the value. The changes of sexual satisfaction scores of the patients and their spouses were observed before and after treatment. The sexual satisfaction scores of the patients were evaluated by 6, 7, and 8 points of the International Erectile Function Index (IIEF), with a total score of 0–15 points. The scores of 10, 13, and 14 in the IIEF table were used to evaluate the spouse's sexual satisfaction with a total score of 0 to 15 points.

### 2.5. Sexual Satisfaction of Spouse

The observation form of spouse satisfaction was filled in. It was recorded once before the treatment, once at the end of the treatment, and follow-up was performed once 3 months after the treatment.

### 2.6. Determination of Serum Testosterone

The serum testosterone level of the selected subjects was measured by ELISA at 8–10 a.m., and the unit was nmol/*L*.

### 2.7. Safety Test

(1) The general physical examination items were checked (once before and after treatment). (2) Possible adverse reactions, such as diarrhea, abdominal pain, and abnormal discomfort of penile skin, were observed, and at the same time, whether women have abnormal discomfort of vagina, etc. was also observed.

### 2.8. Statistical Analysis

All data were analyzed with the SPSS18.0 statistical software. The counting data were analyzed by the chi square test. The measurement data were expressed in (*x* ± *s*), and the difference was statistically significant (*P* < 0.05).

## 3. Results

### 3.1. General Information Comparison

There was no significant difference in the general information between the two groups, which was comparable (*P* > 0.05) (Table 1).

### 3.2. Comparison of IELT and Sexual Life Satisfaction Scores of Patients and Spouses between the Two Groups before and after Treatment

IELT was prolonged in both groups after treatment. At the same time, the IELT of the observation group was 3.28 ± 0.59, which was significantly higher than that of the control group (3.09 ± 0.62) after treatment. The sexual life satisfaction scores of patients and spouses in each group were 10.06 ± 1.28, which was significantly higher than those (6.85 ± 1.02) before treatment (*P* < 0.05). After treatment, the sexual life satisfaction score of patients and spouses in the observation group was 10.86 ± 1.49, which was higher than that (10.57 ± 1.75) in the control group (*P* < 0.05) (Table 2).

### 3.3. Comparison of Serum Testosterone Changes between the Two Groups before and after Treatment

Before treatment, there was no significant difference in serum testosterone levels among all groups (*P* > 0.05). The serum testosterone level after treatment in all groups (13.28 ± 3.15, 15.88 ± 4.71) was decreased compared with that before treatment (26.16 ± 5.26, 25.97 ± 5.58), with statistical significance (*P* < 0.05). After treatment, the level of serum testosterone in the observation group was 13.28 ± 3.15, which decreased significantly compared with the control group 915.88 ± 4.71) (Table 3).

### 3.4. Adverse Reactions

In the observation group, 5 cases had adverse reactions, including 2 cases of dizziness and 3 cases of subcutaneous hematoma. In the control group, there were 6 cases of malady, 4 cases of stomach discomfort, 1 case of mild diarrhea, and 1 case of dizziness.

### 3.5. Security Testing

Before and after treatment, no abnormality was found in blood, urine and stool routine tests, electrocardiogram, and liver and kidney functions in the two groups. After treatment, there were no serious adverse reactions in the two groups, and no patients were terminated due to adverse reactions.

## 4. Discussion

Traditional Chinese medicine believes that the etiology of premature ejaculation is caused by many aspects, which is most closely related to the center of the five Zang organs, liver, and kidney [5]. Its mechanism is in the heart, its movement is in the liver, and it is hidden in the kidney. If the functions of the heart, liver, and kidney are abnormal, such as pouring damp heat into the liver, uncomfortable liver Qi, and liver depression and fire; heart-kidney disharmony and hyperactivity of heart fire; and kidney deficiency, can lead to adverse catharsis, dereliction of duty in sealing and hiding, failure of God, resulting in no right to restrict Jingguan and premature ejaculation due to easy opening of Jingguan. Western medicine believes that the etiology and pathogenesis of this disease are complex, and the specific pathogenesis is inconclusive at present. There are various methods to treat the disease, but no curative effect has been widely recognized. Sertraline hydrochloride, as a highly selective serotonin reuptake inhibitor, can inhibit the reuptake of serotonin in ejaculatory central neurons so as to reduce the excitability of ejaculatory central neurons. On the other hand, sertraline has weak affinity for dopamine receptor, cholinergic receptor, histamine receptor, and adrenergic receptor and will not enhance the activity of catechol neurotransmitters so as to achieve the effect of treating premature ejaculation [6, 7]. However, the drug takes effect 1–2 weeks after taking, often including drowsiness, dry mouth, dizziness, nausea, diarrhea, decreased sexual desire, and nonejaculation [8, 9].

IELT and patient and spouse satisfaction score are commonly used to evaluate the efficacy of premature ejaculation. In this study, the IELT of each group was prolonged after treatment compared with that before treatment, and the difference was statistically significant, indicating that both traditional Chinese medicine and acupuncture had good therapeutic effects in the treatment of premature ejaculation, while electroacupuncture group had better efficacy compared between groups. The results showed that electroacupuncture treatment of premature ejaculation was better than traditional Chinese medicine in IELT and satisfaction score of patient and spouse. The adverse reactions of acupuncture were not significant. Erection is a prerequisite for sexual intercourse, and testosterone plays an important role in erection. Testosterone plays a central and peripheral regulatory role in penile erection response, and a certain level of testosterone is a necessary condition for maintaining sexual desire and penile erection [10]. Corona et al. [11] showed that high serum testosterone level is related to the occurrence of premature ejaculation, and delayed ejaculation is more likely to occur in patients with low serum testosterone. Sakamoto et al. [12] also found that the serum free testosterone level and serum FSH level of patients with premature ejaculation were significantly higher than those of patients without premature ejaculation, but there was no significant difference in the total serum testosterone level between them. In this study, serum testosterone in each group was lower after treatment than before, and the difference was statistically significant. After treatment, the decrease of serum testosterone in the electroacupuncture group was more obvious than that in the traditional Chinese medicine group. It is suggested that electroacupuncture may improve the symptoms of premature ejaculation by reducing the serum testosterone level to some extent. The mechanism of acupuncture in the treatment of premature ejaculation will be further studied in the future.

However, there are also limits in this study. The number of patients is small, which is not so scientific. Besides, the mechanism under this treatment was not clarified, which need further studies to explain it.

## 5. Conclusion

In conclusion, acupuncture therapy based on meridian points has definite curative effect in the treatment of premature ejaculation. Besides, acupuncture is relatively simple, convenient, and easy to implement, with minimal trauma and almost no side effects. Therefore, it is recommended to be popularized and applied in clinical practice. However, due to the small number of patients included in the current study, the overall level of the study is not high, and because there is no unified diagnostic standard and efficacy evaluation standard is inconsistent, the efficacy of each study is prone to bias, resulting in authenticity. Therefore, more researchers and patients need to join the clinical study for further verification.

## Figures and Tables

**Table 1:** General information comparison.

Group	No. of patients (*n*)	Age	Course of disease	No. of cases with different severity before treatment (*n*)		
				Light	Moderate	Severe
Observation group	25	32.68 ± 4.76	39.82 ± 7.95	18	6	1
Control group	25	33.57 ± 5.02	40.07 ± 8.75	17	7	1

**Table 2:** Comparison of IELT and sexual life satisfaction scores of patients and spouses between the two groups before and after treatment.

Item	Time	Observation group	Control group	*P* value
IELT	Before the treatment	1.08 ± 0.36	1.06 ± 0.44	*P* < 0.05
	After the treatment	3.28 ± 0.59	3.09 ± 0.62	

Patient satisfaction score of sexual life	Before the treatment	6.85 ± 1.02	6.91 ± 1.14	*P* < 0.05
	After the treatment	10.06 ± 1.28	9.86 ± 1.67	

Spouse's sexual satisfaction score	Before the treatment	4.85 ± 0.98	4.90 ± 1.04	*P* < 0.05
	After the treatment	10.86 ± 1.49	10.57 ± 1.75	

**Table 3:** Comparison of serum testosterone changes between the two groups before and after treatment.

Item	Time	Observation group	Control group	*P* value
Testosterone level	Before the treatment	26.16 ± 5.26	25.97 ± 5.58	*P* < 0.05
	After the treatment	13.28 ± 3.15	15.88 ± 4.71	

## Data Availability

The data used to support this study are available from the corresponding author upon request.

## References

[1] Althof S. E., Abdo C. H. N., Dean J. (2010). International society for sexual medicine’s guidelines for the diagnosis and treatment of premature ejaculation. *The Journal of Sexual Medicine*.

[2] Xin Z. C., Chung W. S., Choi Y. D., Seong D. H., Choi Y. J., Choi H. K. (1996). Penile sensitivity in patients with primary premature ejaculation. *The Journal of Urology*.

[3] Xin Z. C., Choi Y. D., Seong D. H., Choi H. K. (1995). Sensory evoked potential and effect of SS-cream in premature ejaculation. *Yonsei Medical Journal*.

[4] Waldinger M. D. (2002). The neurobiological approach to premature ejaculation. *The Journal of Urology*.

[5] Waldinger M. D. (2008). Recent advances in the classification, neurobiology and treatment of premature ejaculation. *Sexual Dysfunction*.

[6] Buvat J., Tesfaye F., Rothman M., Rivas D. A., Giuliano F. (2009). Dapoxetine for the treatment of premature ejaculation: results from a randomized, double-blind, placebo-controlled phase 3 trial in 22 countries. *European Urology*.

[7] Mcmahon C. G., Althof S. E., Waldinger M. D. (2008). An evidence-based definition of lifelong premature ejaculation: report of the international society for sexual medicine (ISSM) ad hoc committee for the definition of premature ejaculation. *The Journal of Sexual Medicine*.

[8] Peeters M., Giuliano F. (2008). Central neurophysiology and dopaminergic control of ejaculation. *Neuroscience & Biobehavioral Reviews*.

[9] Donatucci C. F. (2006). Etiology of ejaculation and pathophysiology of premature ejaculation. *The Journal of Sexual Medicine*.

[10] Giuliano F. (2007). 5-hydroxytryptamine in premature ejaculation: opportunities for therapeutic intervention. *Trends in Neurosciences*.

[11] Corona G., Jannini E. A., Mannucci E. (2008). Different testosterone levels are associated with ejaculatory dysfunction. *The Journal of Sexual Medicine*.

[12] Sakamoto H., Takanami K., Zuloaga D. G. (2009). Androgen regulates the sexually dimorphic gastrin-releasing peptide system in the lumbar spinal cord that mediates male sexual function. *Endocrinology*.

